This article has been retracted.

# Effect of Recombinant Netrin-1 Protein Combined with Peripheral Blood Mesenchymal Stem Cells on Angiogenesis in Rats with Arteriosclerosis Obliterans

**DOI:** 10.1155/2022/3361605

**Published:** 2022-07-26

**Authors:** Jie Zeng, Cong Lu, Hui Huang, Jianxin Huang

**Affiliations:** ^1^Department of Cardiology, Sichuan Academy of Medical Sciences & Sichuan Provincial People's Hospital, Chengdu, 610072 Sichuan, China; ^2^Department of Anesthesiology, Sichuan Academy of Medical Sciences & Sichuan Provincial People's Hospital, Chengdu, 610072 Sichuan, China

## Abstract

This work was aimed to explore the effect of recombinant netrin-1 protein and peripheral blood mesenchymal stem cells (MSCs) on the angiogenesis ability of atherosclerosis. 28 Sprague Dawley (SD) rats were taken as research models. The arterial occlusion models were created by surgery and then divided into the saline control group (*n* =7), netrin-1 treatment group (*n* =7), MSCs treatment group (*n* =7), and netrin-1 + MSCs combined treatment group (*n* =7). The peripheral blood MSCs were extracted from the peritoneal cavity of diseased SD rats and cultured alone or in combination with netrin-1. The individually cultured MSCs and netrin-1 were locally injected into the ischemic tissues of SD rats. The Tarlov scoring was performed at the first, second, and third week of treatment, respectively. The expression of vascular endothelial growth factor (VEGF) was also measured by quantitative real-time polymerase chain reaction (qRT-PCR), and the capillary density was measured by immunofluorescence staining. The mean maximum contractility of the gastrocnemius muscle in each group was determined in the third week after treatment. The Tarlov score of the netrin-1 + MSCs group was significantly higher than that of the control group (*P* < 0.05) at the second week. To the 4th week of treatment, the Tarlov score of the netrin-1 + MSCs group was highly increased compared to the netrin-1 group and the MSCs group (*P* < 0.05). The expression of VEGF in the treatment groups was greatly increased each week compared to the control group (*P* < 0.05). Compared with the netrin-1 and the MSCs groups, the VEGF was also notably increased in the netrin-1 + MSCs group (*P* <0.05). The capillary densities of the treatment groups were observably greater than that of the control group in the second and third weeks (*P* <0.05), while the capillary density in the netrin-1 + MSCs group was also significantly increased than those in the netrin-1 group and the MSCs group (*P* < 0.05). The mean maximum contractility of the netrin-1 + MSCs group was remarkably higher than that of the other groups (*P* < 0.05). The netrin-1 + MSCs group achieved the higher Tarlov score, higher VEGF expression, higher capillary density, and better muscle recovery than netrin-1 and MSCs treatments.

## 1. Introduction

Arteriosclerosis obliterans is the embodiment of atherosclerosis in the local region of the limb and is the most common and important type of atherosclerosis [1]. Atherosclerosis obliterans is the precipitation of membrane lipid in some arterial regions, accompanied by the proliferation of smooth muscle cells and fibrous matrix components, which gradually develops into pathological plaques, resulting in insufficient blood supply to the limbs, loss of elasticity of the skin and muscles, and reduced motor ability of the patients' limbs [2]. Smoking, diabetes, hypertension, hyperlipidemia, and excessive obesity are all important causes of atherosclerosis obliterans, and cases mostly appear in middle-aged and elderly male patients [3]. Its course can be divided into four periods: asymptomatic period, intermittent claudication period, rest pain period, and tissue necrosis [4]. Generally, the treatment of arteriosclerosis obliterans consists of nonsurgical treatment and surgical treatment. Nonsurgical treatment includes control of blood pressure, blood sugar, and blood lipids, changing the habit of smoking and drinking, rehabilitation exercise, and drug treatment. Surgical treatment includes traditional open bypass surgery and minimally invasive surgery. The therapeutic effect of surgical treatment is good, but attention should be paid to the occurrence of stenosis. If the disease is not treated in time, it will face the risk of amputation or even death [5].

Mesenchymal stem cells (MSCs) are a kind of human stem cells derived from the mesoderm in the early stage of development. It can differentiate into myocardial, nerve, endothelial, muscle, and other tissue cells under inductions. It still has differentiation potential after continuous culture in vitro and plays an important role in the treatment of cardiovascular and cerebrovascular diseases, nervous system diseases, and immune system diseases [6–9]. At present, MSCs can be obtained from various tissues such as umbilical cord blood, bone marrow, muscle, amniotic fluid, peripheral blood, and adipose tissue [10], which do not increase the amputation rate and mortality rate after transplantation into patients with atherosclerosis obliterans after culture, and its pro-angiogenic effect is irreplaceable by other treatment modalities [11].

Netrin-1 protein is a soluble neural guidance factor first discovered in vertebrates. It is an unstable and hydrophilic alkaline secreted protein with a random coiled secondary structure. It is a member of the Netrin protein family, having strong chemical induction ability to promote axon extension, in addition to regulating cell migration, motility, proliferation, and other effects [12, 13]. In recent years, some scholars have found that netrin-1 protein not only plays a role in the nervous system but also plays a great role in promoting angiogenesis [14, 15]. Netrin-1 has been revealed to be a potent angiogenic growth factor and potentiates vascular endothelial growth factor (VEGF) responses [16].

The model of the atherosclerosis obliterans rat by artificial culture was established. The MSCs extracted from the peripheral blood of the abdominal aorta of the rat were cultured and expanded in vitro. The MSCs cultured with netrin-1 protein were transplanted into the ischemic tissue of rat limbs. The recovery of ischemic tissue was observed and scored. The expression of vascular intradermal growth factor, the vascular density of ischemic tissue, and the average maximum contraction rate of gastrocnemius muscle of ischemic tissue were determined.

## 2. Experimental Methods

### 2.1. Materials and Methods

This experiment was approved by the Ethics Committee of the hospital; after that, the research was started. 28 male healthy Sprague Dawley (SD) rats (16 months old, 310 ± 10 g, and specific-pathogen-free) were provided by the XX Laboratory Animal Center. These rats were fed with animal fat and other high-fat diet for 6 weeks, then they were randomly divided into 4 groups, with 7 rats in each group. The groups were the netrin-1 + MSCs combined treatment group, the netrin-1 treatment group, the MSCs treatment group, and the normal saline group (blank control).

### 2.2. Model Making

The model of arteriosclerosis obliterans rats was established. From the third day of feeding, rats were subcutaneously injected with granulocyte colony-stimulating factor at a dose of 50 *μ*g/1,000 g to stimulate bone marrow to produce granulocytes and stem cells and release them into the blood. Rats were anesthetized with 2% sodium pentobarbital at a dose of 30 mg/kg under sterile conditions. The hind limbs and abdomen were routinely performed for skin preparation and disinfection. The skin and subcutaneous tissue were cut to reveal the left femoral artery. The branches were ligated. The anterior wall of femoral artery was cut and implanted with appropriate anticoagulant silicone tube. The incision was sutured after fixation of tube. 2 mL arterial blood was extracted from abdominal aorta and put into heparin anticoagulant tube, the wound of rats was sutured, and disinfection was carried out. The postoperative feeding methods of rats were the same as before.

### 2.3. Culture and Detection of Peripheral Blood MSCs

#### 2.3.1. Culture of Peripheral Blood MSCs

The obtained abdominal aortic blood was cultured, and only the netrin-1 + MSCs combined treatment group and MSCs treatment group were isolated and cultured. The collected peripheral blood was diluted with phosphate buffer solution at a volume ratio of 1 : 1, introduced into a centrifuge tube, and added with 1.077 g/L Percoll cell separation solution. The solution was centrifuged at a rate of 2,000 r/min for 20 minutes. After centrifugation and stratification, the first layer was discarded with a pipette. The second layer of cells was collected and transferred to a culture flask. DMEM/F12 medium containing 10% fetal bovine serum was added to performed observation at 37°C. When the peripheral blood MSCs grew and fused to more than 80%, they were transferred for subculture.

#### 2.3.2. Detection of MSCs

The subcultured MSCs were treated with 0.25 g trypsin for 5 min and centrifuged for 5 min. The cell pellets were collected and washed three times with phosphate-buffered saline solution. 25 *μ*L of monoclonal antibodies were added to detect the surface markers CD44, CD90, and CD105 of highly expressed MSCs and the surface markers CD34 and CD45 of lowly expressed MSCs, which were then identified by flow cytometry (CytoFL EX, Beckman Coulter Inc.).

### 2.4. Transplant Therapy

#### 2.4.1. Transplant Method

On the day of treatment, netrin-1 + MSCs group of rats was intramuscularly injected with 1 × 10^6^ stem cells and 1 *μ*g netrin-1 in the left hind limb, stem cells group of rats was intramuscularly injected with 1 × 10^6^ stem cells in the left hind limb, netrin-1 group of rats was intramuscularly injected with 1 *μ*g netrin-1 in the left hind limb, and the control group of rats was intramuscularly injected with 0.3 mL 0.9% sodium chloride injection in the left hind limb. Six points were selected as injection points on the left hind limb.

#### 2.4.2. Tarlov Score after Treatment

Animals in the four groups underwent Tarlov scoring during the first, second, and third weeks of treatment. The scoring criteria are as follows (Table 1).

### 2.5. Determination of VEGF Expression

VEGF was measured in the four groups of rats at weeks 1, 2, and 3 of injection therapy.

The method is as follows.

1. RNA extraction from rat gastrocnemius muscle

Rat gastrocnemius muscle was taken and liquid nitrogen was added to grind for 3 times, Trizol reagent was added after homogenization to further break up the cell components, then it was extracted with chloroform, and the aqueous phase and organic phase were separated after centrifugation. The aqueous phase was precipitated with isopropanol to obtain RNA, 1 *μ*L of sample was taken and diluted to 100 times to determine the RNA concentration and absorbance OD260/280 ratio. It was stored at -75°C in an ultra-low temperature freezer after passing the determination.

(2) Reverse transcription to cDNA

Reverse transcriptase was inactivated using TAKARA RR047A reverse transcription kit at a reverse transcription temperature of 37°C for 30 minutes and a reaction at 85°C for 10 seconds after completion of transcription.

(3) Primer design and quantitative detection of quantitative real-time polymerase chain reaction (qRT-PCR)

According to the mRNA sequence analysis result of VEGF, the upstream primer was designed as 5′-CCTGGCTTTACTGCTCTACCT-3′, while the downstream primer was the specific primer of 5′-GATGTCCACCAGGGTCTCAAT-3′. *β*-Actin was used as an internal reference, then the upstream primer was 5′-TCAGGTCATCACTATCGGCAAT-3′, and the downstream primer was 5′-AAAGAAAGGGTGTAAAACGCA-3′. SYBR®Premix Ex TaqTM (TIi RNaseH Plus) fluorescence quantitative kit of Takara Bio Inc. was adopted for qRT-PCR, and the Ct value of each sample was recorded.

(4) Determination of VEGF

The 2^-△△CT^ method was used to compare the expression of VEGF in the gastrocnemius muscle of treated and untreated rats in each group.

### 2.6. Determination of Capillary Density

The gastrocnemius muscle specimens were prepared as follows. The rat gastrocnemius muscle was taken, fixed with 4% paraformaldehyde solution, dehydrated with different concentrations of alcohol, vitrified with xylene, embedded with a paraffin embedding machine (Leica Biosystems Nussloch GmbH), and sliced with a microtome (Leica Biosystems Nussloch GmbH). As fluorescently labeled fluorescein isothiocyanate solution was added, the slices reacted at 5°C for 8 hours. Then, the specimens were observed using an inverted fluorescence microscope and counted capillary density using SlideBook software.

### 2.7. Determination of Maximum Contractility of Gastrocnemius Muscle

The mean maximum isometric contractility of the gastrocnemius muscle of rats in the four groups was measured in the third week of treatment using a bio-signal acquisition system. The models were the sciatic nerve-gastrocnemius muscle models. Stimulating electrodes were utilized to stimulate the sciatic nerve of rats surgically dissected out under anesthesia. The distal end of the tendon was connected with a tension sensor, and the stimulation frequency was appropriately increased to make the gastrocnemius muscle contract strongly. Then, the maximum isometric contractility of the gastrocnemius muscle of rats could be measured.

### 2.8. Data Processing Method

All experimental results were expressed in the form of mean combined with error, and SPSS 24.0 was used to process the data. Independent samples were analyzed by *t*-test, and comparisons of results among multiple groups required the *F* test. *P* > 0.05 indicated no statistically significant difference, and *P* < 0.05 indicated statistically significant difference.

## 3. Experimental Results

### 3.1. Primary and Subculture Results of Peripheral Blood MSCs

#### 3.1.1. Observation Results under Inverted Microscope

During the primary culture of MSCs, adherent growth appeared in about 24 hours, and the cells were round, spindle-shaped, or triangular, and they grew slowly (Figure 1(a)). After the medium was changed, the cells proliferated obviously and manifested in various forms, mainly in the shape of spindle (Figure 1(b)). After 12 days, 70%-80% of the cells were fused and reached the subculture standard. The subcultured cells were single in morphology, which were spindle-shaped or flat (Figure 1(c)). The cells swirled and radially arranged when they proliferated to cell fusion (Figure 1(d)).

#### 3.1.2. Identification of Surface Markers of Hematopoietic Stem Cells by Flow Cytometry

After identification by flow cytometry, the surface markers CD44, CD90, and CD105 of peripheral blood MSCs were highly expressed, and the expression rates were 96.7%, 98.4%, and 97.5%, respectively. The expression rates of hematopoietic stem cell surface markers CD34 and CD45 were low, which were 0.15% and 0.11%, respectively. The results are listed in Table 2.

### 3.2. Tarlov Scoring Results after Treatment

During the experiment, no rats died. In the first week of treatment, the Tarlov score was 2.1 ± 0.3 in the control group, 2.15 ± 0.4 in the netrin-1 group, 2.13 ± 0.5 in the MSCs group, and 2.2 ± 0.4 in the netrin-1 + MSCs group. There was no significant difference among the groups (*P* > 0.05). In the second week of treatment, the Tarlov score was 2.15 ± 0.6, 2.2 ± 0.5, 2.3 ± 0.5, and 2.5 ± 0.2 in the control, netrin-1, MSCs, and netrin-1 + MSCs groups, respectively. Compared with the control group, that of the netrin-1 + MSCs group increased greatly (*P* < 0.05). In the third week of treatment, Tarlov score was 2.1 ± 0.6, 2.7 ± 0.4, 3.1 ± 0.5, and 3.9 ± 0.5 in the control, netrin-1, MSCs, and netrin-1 + MSCs groups, respectively. The Tarlov scores of the netrin-1, MSCs, and netrin-1 + MSCs groups were considerably increased compared to the control group in the third week (*P* < 0.05). Meanwhile, the Tarlov score of the netrin-1 + MSCs group was also notably higher than those of the netrin-1 and the MSCs groups (*P* < 0.05). All these details are shown in Figure 2.

### 3.3. Expression of VEGF

The expression levels of VEGF in the ischemic tissues of the four groups of rats were evaluated by qRT-PCR, as shown in Figure 2, that in each group was compared with the control group. In the first week, the expression levels in the netrin-1, MSCs, and netrin-1 + MSCs groups were 1.2 times, 1.3 times, and 1.4 times that of the control group, respectively. In the second week, the expression levels of netrin-1 group and MSCs group were 1.3 times and 1.2 times that of the control group, respectively. The expression level of the netrin-1 + MSCs group was 1.45 times that of the control group. In the third week, the expression levels of netrin-1 and MSCs groups were 1.15 times and 1.2 times that of the control group, while that of the netrin-1 + MSCs group reached 1.3 times that of the control group. The expression level of VEGF in the netrin-1 + MSCs group was always markedly higher than that in the other groups in the first, second, and third weeks (*P* < 0.05). The expression level of VEGF was not significantly different between netrin-1 group and MSCs group (*P* > 0.05), but it was also observably higher than that in the control group (*P* < 0.05). The detailed comparisons are shown in Figure 3.

### 3.4. Capillary Densitometry Results

Figures 4(a)–4(d) display the observed capillary images (×400). From the images, the control group showed the least capillaries (Figure 4(a)), followed by the netrin-1 group and the MSCs group (Figures 4(b) and 4(c)), and the netrin-1 + MSCs group had the most (Figure 4(d)). As shown in Figure 4(e), in the first week of treatment, the mean capillary density was 286 ± 26 mm^2^ in the control group, 291 ± 17 mm^2^ in the netrin-1 group, 293 ± 23 mm^2^ in the MSCs group, and 284 ± 17 mm^2^ in the netrin-1 + MSCs group. There was no remarkable difference among the groups in the first week (*P* > 0.05). In the second week, the mean capillary density was 288 ± 17 mm^2^, 413 ± 23 mm^2^, 399 ± 16 mm^2^, and 421 ± 25 mm^2^ in the control, netrin-1, MSCs, and netrin-1 + MSCs groups, respectively. Compared to the control group, the difference from each group was quite significant (*P* < 0.05). In the third week of treatment, the mean capillary density was 289 ± 14 mm^2^, 520 ± 21 mm^2^, 539 ± 14 mm^2^, and 601 ± 32 mm^2^ in the control, netrin-1, MSCs, and netrin-1 + MSCs groups, respectively. In contrast to the control group, the capillary density increased greatly in each group (*P* < 0.05). The capillary density in the netrin-1 + MSCs group was obviously higher than that in the netrin-1 group and MSCs group (*P* < 0.05).

### 3.5. Maximum Contractility of Gastrocnemius Muscle Results

After three weeks of treatment, the mean maximum contractility of the control, netrin-1, MSCs, and netrin-1 + MSCs groups was 0.51 ± 0.30 N, 0.61 ± 0.35 N, 0.62 ± 0.37 N, and 0.65 ± 0.35 N, respectively. Among them, the mean maximum contractility of the netrin-1 + MSCs combination group was significantly higher than that of the other groups, which indicated that the combination therapy had the best effect on muscle recovery in rats with arteriosclerosis obliterans and meant that the ischemic tissue was better recovered (Table 3).

## 4. Discussion

In this experiment, it simulated the transplantation process of autologous peripheral blood cells in patients with arteriosclerosis obliterans through a rat model to investigate the effect of angiogenesis [17, 18]. The role of stem cells and netrin-1 has been analyzed in animal models of acute ischemia, which can be made easily by removing the femoral artery, so acute ischemia models are easy to make [19]. However, acute ischemia can lead to fierce body response, significant inflammatory effect, and affect the expression of VEGF. At present, scholars have explored the extraction of stem cells from umbilical cord blood for transplantation in the treatment of arteriosclerosis obliterans, and found that the angiogenesis ability of patients has been improved, and the corresponding results can also be obtained in this experiment [20]. The animal model of chronic limb ischemia was created by feeding rats with food and artificial surgical implantation, which could better simulate the pathogenesis of peripheral vascular disease [21].

Tarlov scoring is the motion evaluation criteria proposed by Tarlov in 1953 for animals after spinal compression injury. It has been widely used after being improved by scholars [22]. The Tarlov scores of the netrin-1 group, the MSCs group, and the netrin-1 + MSCs group were not statistically different in the first week of this research. In the second week, the Tarlov score of the netrin-1 + MSCs group was observably higher than that of the control group, indicating that the combined treatment method could exert its effect faster than only using netrin-1 or MSCs alone. In the third week, the Tarlov score of netrin-1 + MSCs group was greatly higher than the control, the netrin-1, and the MSCs groups. This suggested that with the prolongation of the treatment time, the treatments all worked; but in general, the netrin-1 + MSCs was superior to the single use of netrin-1 or MSCs. Besides, in the observation of SD rats, it was found that the rats treated with the combination could recover to the state of standing and slow movement after three weeks of treatment. The expression of VEGF was relatively close to the Tarlov score, which perhaps explains why the combined treatment of netrin-1 + MSCs was more effective. The expression level of VEGF was always significantly the highest in the combined treatment of netrin-1 + MSCs at any stage of the experiment. To further confirm the experimental results, the capillary density of the tissue and the maximum contractility of the gastrocnemius muscle in the third week were measured in this research. The results were close to the performance of VEGF. The capillary density was greatest in the netrin-1 + MSCs group, while the mean gastrocnemius contractility measured at the third week was also the greatest. The increased capillary density suggested that the angiogenesis ability of the rats was well restored, and the therapeutic effect was good. The greater the maximum contractility of the gastrocnemius muscle demonstrated that the blood supply to the muscle was guaranteed due to the vascular permeability, and the muscle function was restored.

## 5. Conclusion

Culture and recombination of netrin-1 with peripheral blood MSCs significantly improved the therapeutic effect of transplantation, especially in the third week, and treated rats were able to obtain higher Tarlov scores compared with other groups, with higher expression of vascular intradermal growth factor, greater capillary density of ischemic tissue, and best muscle recovery. This experiment provides a good idea for the clinical treatment of arteriosclerosis obliterans. However, the sample size was small, and only a single disease was taken into consideration, as diabetes, neurological diseases, hypertension, and other possible diseases were not considered. Thus, the safety and effectiveness of its role on other diseases in the clinical practice needed to be further studied.

## Figures and Tables

**Figure 1:** Observation picture under inverted microscope (×400). Note: Figure 1(a) shows the cell morphology at the initial stage of inoculation, Figure 1(b) shows after medium exchange culture, Figure 1(c) shows at the initial stage of subculture, and Figure 1(d) shows at the second generation of subculture.

**Figure 2:** Tarlov score of each group at the first week, the second week, and the third week after treatment.Note: ∗, #, and ^ indicated a statistically significant difference compared to the control group (*P* < 0.05), the netrin-1 group (*P* < 0.01), and the MSCs group (*P* < 0.01), respectively.

**Figure 3:** Expression level of VEGF at the first week, the second week, and the third week after treatment.Note: ∗ indicated a statistically significant difference compared to the control group (*P* < 0.05); # marked a statistical difference compared to the netrin-1 group (*P* < 0.01); and ^ indicated a statistical difference as well compared to the MSCs group (*P* < 0.01).

**Figure 4:** Capillary density at the first week, the second week, and the third week after treatment. Note: ∗, #, and ^ indicated the statistically significant differences in comparison with the control group (*P* < 0.05), the netrin-1 group (*P* < 0.01), and the MSCs group (*P* < 0.01), respectively.

**Table 1:** Tarlov scoring criteria.

Content	Score
The lower extremities are completely paralyzed	0
Perceptible movement of the lower extremities joints	1
The lower limbs can move freely, but they cannot stand	2
Can stand but cannot walk	3
Lower limb motor function is fully restored and can walk normally	4

**Table 2:** Identification results of surface markers with high and low expression of peripheral blood MSCs.

Groups	Highly expressed MSCs			Low expression of MSCs	
	CD44	CD90	CD105	CD34	CD45
Expression rate	96.7%	98.4%	97.5%	0.15%	0.11%

**Table 3:** Measurement results of maximum contractility of gastrocnemius muscle in each group at the third week.

Groups	Control group	Netrin-1 group	MSCs group	Netrin-1 + MSCs group
Muscular strength (N)	0.51 ± 0.32	0.61 ± 0.35∗	0.62 ± 0.37∗	0.65 ± 0.35∗#^

Note: ∗ marked a statistically significant difference compared to the control group (*P* <0.05), # indicated that compared to the netrin-1 group (*P* <0.01), and ^ indicated that compared to the MSCs group (*P* <0.01).

## Data Availability

All data, models, and code generated or used during the study appear in the submitted article.
